The article "Demographics and Economic Burden of Nasopharyngeal Carcinoma Inpatients" was retracted in 2023. Reasons: signs of a paper mill; compromised peer review; unreliable results or conclusions.

# Demographics and Economic Burden of Nasopharyngeal Carcinoma Inpatients

**DOI:** 10.1155/2022/6958806

**Published:** 2022-06-15

**Authors:** Dong Yang, Nengfu Bin, Ziyan Zhou, Zhiru Li, Mingjun Shen, Chaolin Yang, Yating Qin, Rensheng Wang, Wei Lv, Bo Wei, Lifang Zhou, Min Kang

**Affiliations:** ^1^Department of Radiation Oncology, The First Affiliated Hospital of Guangxi Medical University, Nanning, 530021, Guangxi, China; ^2^The First Affiliated Hospital, Department of Radiation Oncology, Hengyang Medical School, University of South China, Hengyang, 421001 Hunan, China; ^3^Key Laboratory of Early Prevention and Treatment for Regional High Frequency Tumor (Guangxi Medical University), Ministry of Education, Nanning, 530021 Guangxi, China; ^4^Guangxi Key Laboratory of Immunology and Metabolism for Liver Diseases, Nanning, 530021 Guangxi, China; ^5^Health Statistics information Center of Guangxi Zhuang Autonomous Region, Nanning, 530021 Guangxi, China; ^6^Guangxi Medical University Cancer Hospital, Nanning 530021, Guangxi, China; ^7^The Fourth Affiliated Hospital of Guangxi Medical University, Liuzhou 545005, Guangxi, China; ^8^Liuzhou Center for Disease Prevention and Control, Liuzhou 545005, Guangxi, China

## Abstract

**Objective:**

Nasopharyngeal carcinoma is particularly prevalent in Guangdong and Guangxi (southern China); the economic burden of nasopharyngeal cancer patients is heavy in China. This study is aimed at retrospectively analyzing the basic features and economic burden of newly diagnosed nasopharyngeal carcinoma patients admitted to the First Affiliated Hospital of Guangxi Medical University and at providing a scientific basis for nasopharyngeal carcinoma prevention and control strategies.

**Methods:**

The data of 3,727 nasopharyngeal carcinoma inpatients diagnosed from January 2012 to December 2020 were extracted from the Guangxi Nasopharyngeal Carcinoma Healthcare Big Data Management Information Platform. Basic demographic characteristics, duration of hospital stay, and hospitalization cost of nasopharyngeal carcinoma patients were collected and analyzed statistically.

**Results:**

The incidence period of nasopharyngeal carcinoma was primarily from 30 to 69 years of age, with the 40–49-year age group comprising the largest proportion of nasopharyngeal carcinoma patients, accounting for 34.18% of the patients with newly diagnosed nasopharyngeal carcinoma in the hospital. The male-to-female ratio was 2.87 : 1. There were 2,223 cases from rural areas, 2,153 from the Han ethnic group, and 1,460 from the Zhuang ethnic group, accounting for 59.65%, 55.77%, and 39.17% of the total number of cases, respectively. The average duration of hospitalization decreased whereas the average hospitalization cost increased annually. Multivariate analysis of hospitalization cost showed that the duration of hospital stay, rural/urban, and ethnicity was the main influencing factors: the longer the duration of hospital stay, the higher the hospitalization cost; patients from rural incurred lower costs than from urban; ethnic Zhuang patients incurred significantly lower costs than patients from other ethnicities.

The article "Demographics and Economic Burden of Nasopharyngeal Carcinoma Inpatients" was retracted in 2023. Reasons: signs of a paper mill; compromised peer review; unreliable results or conclusions.

**Conclusion:**

Early diagnosis and treatment should be actively carried out to reduce the incidence of nasopharyngeal carcinoma, especially for rural, ethnic Zhuang, and males in the 40–49-year age group patients. The future research on nasopharyngeal carcinoma will focus on exploring the pathogenesis of nasopharyngeal carcinoma, improving the screening system, and reducing the burden on patients, in order to further improve the survival rate and quality of life of patients with nasopharyngeal carcinoma.

## 1. Introduction

Nasopharyngeal carcinoma is a malignant tumor originating from the mucosal epithelium of the nasopharynx, which primarily occurs in Southeast Asian countries and southern China. According to the World Health Organization (WHO) International Agency for Research on Cancer, there were 133,000 new nasopharyngeal carcinoma cases and 80,000 deaths worldwide in 2020, including 62,000 new cases and 34,000 deaths in China, accounting for more than 43% of the global disease burden [1]. Nasopharyngeal carcinoma is particularly prevalent in Guangdong and Guangxi (southern China), and the incidence decreases from south to north [2]. The incidence is higher in males than in females, with a ratio of about 2.5 : 1 in China [3, 4]. Moreover, it increases with age in people over 20 years old and reaches its peak at approximately 45 to 60 years old [5]. The etiology of nasopharyngeal carcinoma may be heredity, environmental, and/or linked to Epstein-Barr virus infection [5]. With the development of medical technology, the incidence and mortality of nasopharyngeal cancer in China have decreased significantly compared with the past. However, with the aging of China's population, nasopharyngeal carcinoma incidence and mortality may continue to rise. The incidence of nasopharyngeal cancer in rural residents was significantly higher than that in urban residents (1.5 : 1), especially in males [6]. The economic burden of nasopharyngeal cancer patients presented disparity in different rural and urban areas and showed temporal change; the cancer burden in China remains at a high level despite improvements in health care and increasing funding on cancer control [7]. Data released in 2020 showed that the incidence of nasopharyngeal cancer in Guangxi was 10.71/100,000, and the mortality was 5.15/100,000, significantly higher than the national level (2.67/100,000 and 1.31/100,000); this shows that the incidence and mortality of nasopharyngeal cancer in Guangxi are still higher than the national level [8]. Increasing disease burden on patients and their families will worsen prevention and control.

The article "Demographics and Economic Burden of Nasopharyngeal Carcinoma Inpatients" was retracted in 2023. Reasons: signs of a paper mill; compromised peer review; unreliable results or conclusions.

This study is aimed at retrospectively analyzing the demographics and economic burden of newly diagnosed nasopharyngeal carcinoma patients admitted to the First Affiliated Hospital of Guangxi Medical University in Nanning city from 2012 to 2020 to provide a scientific basis for the formulation of prevention and control strategies.

## 2. Material and Methods

### 2.1. Data Source

We extracted 3,830 cases of nasopharyngeal cancer patients hospitalized and diagnosed in the First Affiliated Hospital of Guangxi Medical University in Nanning city from January 2012 to December 2020 from the Guangxi Nasopharyngeal Carcinoma Healthcare Big Data Management Information Platform. Sample inclusion criteria included (1) medical records with primary diagnosis of nasopharyngeal malignant tumor (ICD-10 disease code C11) after discharge and (2) period of admission from 1 January 2012 to 31 December 2020. The general information of the patients (gender, age, address, ethnic origin, regional origin, and medical insurance payment category), their duration of hospitalization, total hospitalization cost, and other information were extracted. Sample exclusion criteria included (1) cases with hospitalization of <1 day, (2) incomplete patient information, and (3) cases with other complications. The resulting cohort included 3727 participants for the final analysis (Figure 1). The study was approved by the ethics review board of the First Affiliated Hospital of Guangxi Medical University (2021-102).

### 2.2. Statistical Analysis

The data collected were entered into a Microsoft Excel spreadsheet and statistically analyzed (IBM SPSS Version 26; International Business Machine, Armonk, NY, United States of America). Qualitative data were statistically described by frequency and composition ratio; the *χ*^2^ test was used for comparison between groups, and the rank-sum test was used for statistical analysis of different types of data. The Mann–Whitney *U* test was used for the influence of gender and rural/urban on total hospitalization cost. The Kruskal-Wallis *H* test was used for the influence of ethnicity on total hospitalization costs. Spearman rank correlation analysis was used to assess the influence of age and duration of stay on total hospitalization cost. A multiple linear regression model was used to analyze the factors influencing hospitalization expenses. *P* values < 0.05 were considered statistically significant. *P* values ≤ 0.001 were considered statistically significant highly.

The article "Demographics and Economic Burden of Nasopharyngeal Carcinoma Inpatients" was retracted in 2023. Reasons: signs of a paper mill; compromised peer review; unreliable results or conclusions.

## 3. Results

### 3.1. Demographic Characteristics

From 2012 to 2020, a total of 3,727 nasopharyngeal cancer patients were diagnosed, including 2,765 males and 962 females, with a male-to-female ratio of 2.87 : 1. The number of cases was highest in 2017 (504 cases), and the male-to-female ratio was highest in 2015 (3.41 : 1), as shown in Table 1. There was no significant difference in gender in different years (*χ*^2^ = 5.655, *P* = 0.686).

Among the 3,727 patients included, the mean age of onset was 46.54 ± 11.26 years, with the youngest being 11 years old and the oldest being 81 years old. The incidence of the disease was primarily concentrated in 30-69-year-old patients, and 40-49-year-old patients accounted for the largest proportion (34.18%). There was no significant difference in gender in the different age groups (*χ*^2^ = 10.795, *P* = 0.148), as shown in Table 2.

Among the 3,727 patients, 938 were from Nanning city, accounting for 25.17% of the total, and 2,789 were from outside Nanning city, accounting for 74.83% of the total. There were 2,223 cases from rural areas, accounting for 59.65% of the total, and 1,504 cases from urban areas, accounting for 40.35% of the total. These data indicate that the incidence of nasopharyngeal carcinoma outside of Nanning is higher than that within Nanning, with rural areas experiencing higher rates than urban areas.

In this study, there were 2,153 (55.77%) patients of Han ethnicity, 1,460 (39.17%) of Zhuang ethnicity, and 114 (3.06%) from other ethnic groups, as shown in Figure 2.

### 3.2. Economic Burden

The average duration of stay of nasopharyngeal cancer patients showed a decreasing trend, with an average annual decrease rate of 3.3% and a month-on-month decrease of 2.5% (Table 3). The average hospitalization cost showed an increasing trend, with an annual average growth rate of 5.9% and a month-on-month increase of 7.5% (Table 4).

### 3.3. Factors Influencing Total Hospitalization Cost

Data from our study show a skewed distribution of the total hospitalization cost; therefore, a nonparametric test (the rank-sum test) was used for statistical analysis.

#### 3.3.1. Relationship between Gender and Total Hospitalization Cost

The median total hospitalization cost for male patients was 77,305.90 yuan, and that for female patients was 76,470.07 yuan, which was not statistically significant (Mann–Whitney *U* test, *Z* = –0.244, *P* = 0.807). Thus, gender was not associated with total hospitalization costs (Table 5).

The article "Demographics and Economic Burden of Nasopharyngeal Carcinoma Inpatients" was retracted in 2023. Reasons: signs of a paper mill; compromised peer review; unreliable results or conclusions.

#### 3.3.2. Relationship between Age and Total Hospitalization Cost

According to the Spearman rank correlation calculation (*R* = –0.003, *P* = 0.8600), there was no correlation between age and total hospitalization cost (Figure 3(a)).

#### 3.3.3. Relationship between Ethnicity and Total Hospitalization Cost

The average hospitalization cost for ethnic Han patients was 68,800.63 yuan, that for ethnic Zhuang patients was 60,624.60 yuan, and that for other patients was 68,787.48 yuan. The nonparametric rank-sum test (Kruskal–Wallis *H* test, *H* = 27.42, *P* ≤ 0.001) suggested that the total hospitalization costs of different ethnic groups were significantly different. After pair-wise comparison, the total hospitalization cost was found to be different between ethnic Han and ethnic Zhuang patients (adjusted *P* ≤ 0.001). There was no difference in total hospitalization cost between Han and other ethnic groups and between Zhuang and other ethnic groups (adjusted *P* = 1.000 and *P* = 1.000, respectively; Table 5).

#### 3.3.4. Relationship between Rural/Urban and Total Hospitalization Cost

The median total hospitalization cost of rural patients was 61,454.37 yuan, and that of urban patients was 71,720.99 yuan. According to the Mann–Whitney *U* test (*Z* = −6.211, *P* ≤ 0.001), the difference was statistically significant. Therefore, it can be assumed that the total cost of hospitalization differs between rural and urban patients (Table 5).

#### 3.3.5. Relationship between Duration of Stay and Total Hospitalization Cost

Spearman rank correlation analysis of the duration of stay and total hospitalization cost (*R* = 0.694, *P* ≤ 0.001) suggested a positive linear correlation; the longer the stay, the higher the cost of hospitalization (Figure 3(b)).

#### 3.3.6. Multivariate Regression Analysis of Total Hospitalization Cost

Since the distribution of hospitalization cost was positively skewed, it presented an approximately normal distribution after logarithmic transformation. Multiple linear regression was performed using hospitalization cost as the dependent variable and ethnicity, rural/urban, and duration of hospitalization as the independent variables. The results showed that the main factors influencing patient hospitalization costs were duration of stay, ethnicity, and rural/urban, as shown in Table 6.

Subgroup multiple linear regression analysis of the impact of rural/urban on total hospitalization costs showed that the total hospitalization costs of rural patients were significantly lower than those of urban patients (*P* ≤ 0.001), as shown in Table 7.

Further analysis of ethnic subgroups using multivariate linear regression analysis showed that total hospitalization expenses for ethnic Zhuang patients were lower than those for ethnic Han patients and other ethnicities (*P* ≤ 0.001 and *P* = 0.039, respectively). Compared with the total cost for patients from other ethnic groups, total costs for Han patients in the hospital showed no significant difference (*P* = 0.823).

The article "Demographics and Economic Burden of Nasopharyngeal Carcinoma Inpatients" was retracted in 2023. Reasons: signs of a paper mill; compromised peer review; unreliable results or conclusions.

## 4. Discussion

At present, the cause of nasopharyngeal cancer is not clear, which increases the difficulty of primary prevention. Moreover, the onset of nasopharyngeal cancer is insidious, and there are no distinct symptoms and signs at the early stage, which complicates secondary prevention. When a patient is diagnosed, they have usually reached the middle and late stages of cancer and face treatment complications, such as a long treatment cycle, poor prognosis, high recurrence rate, and probability of distant metastasis [9, 10]. Hence, improved early diagnosis and treatment and reduced disease burden of nasopharyngeal cancer have become an urgent and critical necessity. The incidence of nasopharyngeal cancer has always been high in southern China [2]. As the largest grade A tertiary hospital in Guangxi Province, the nasopharyngeal cancer cases provided in this study have certain research and reference significance.

A total of 3,727 patients were included in this study. The results show that the onset of nasopharyngeal carcinoma is primarily between 30 and 69 years of age, and that the 40–49-year-old age group represents the largest proportion (34.18% of new cases of nasopharyngeal carcinoma in the hospital). Li et al. [11] analyzed nasopharyngeal carcinoma cases in the Guangxi Tumor Hospital from 2002 to 2011 and showed that the peak age of incidence was in the 41–60-year-old group, accounting for 61.59%. The present study suggests that the age of nasopharyngeal carcinoma has decreased. In all age groups, male patients outnumbered female patients; the male-to-female ratio was 2.87 : 1, which is similar to data in the relevant literature [11]. This suggests that male patients have a heavier disease burden. The male-female ratio also widens with age, primarily owing to differences in social functions between men and women, with men exposed to higher stress environments and other risk factors (such as smoking and work stress) [12]. As such, governments should take gender into account when planning and allocating health resources. The data showed that males aged 30 to 69 are at the highest risk of nasopharyngeal cancer, and screening and protection of this group should be strengthened for the prevention and treatment of nasopharyngeal cancer.

We identified 2,223 cases from rural areas, accounting for 59.65% of the total. Some urban areas of Guangxi Zhuang Autonomous Region are highly industrialized, and some industries have moved to the suburbs and closer to the countryside, resulting in the deterioration of air quality in residential areas. Local residents are easily exposed to harmful substances, increasing disease incidence. In terms of ethnic groups, there were 2,153 ethnic Han patients (55.77%) and 1,460 ethnic Zhuang patients (39.17%), according to the 2017 Guangxi Statistical Yearbook [13]. By the end of 2016, the Han population of Guangxi Zhuang Autonomous Region accounted for 62.8% of the population of Guangxi, whereas the Zhuang population accounted for 31.39%. Zhuang is the most populous ethnic minority in China, most of which live in Guangxi. The distribution of Zhuang population is an important factor affecting the proportion of ethnic population and cancer incidence in Guangxi [14]. The proportion of Zhuang patients in this study was slightly higher, which may be related to the fact that Nanning and its surrounding cities and counties, including Liuzhou, Baise, Laibin, Hechi, and Chongzuo, are inhabited by ethnic Zhuang residents.

The article "Demographics and Economic Burden of Nasopharyngeal Carcinoma Inpatients" was retracted in 2023. Reasons: signs of a paper mill; compromised peer review; unreliable results or conclusions.

High medical expenses are the key factor leading to “high and difficult medical treatment” for ordinary people [15]. Therefore, the key to solving the problem of excessive rise in medical expenses is to control the unreasonable growth of hospitalization expenses. It is particularly important to study and analyze hospitalization expenses and influencing factors. In this study, the average duration of hospitalization of newly diagnosed nasopharyngeal carcinoma patients decreased every year, and this decrease was related to adjusted medical insurance policies [16]. However, the average hospitalization cost increased. In recent years, owing to factors such as the increase in population, price inflation, and medical advancements, medical expenses have also increased year-on-year [17]. Thus, the economic burden of nasopharyngeal cancer is increasing.

Multivariate analysis of hospitalization cost showed that the duration of stay, rural/urban, and ethnicity were the main influencing factors. The duration of stay greatly influenced hospitalization cost: the longer the duration, the higher the cost. To ensure the quality of medical services, the average duration of hospital stay must be shortened [18]; this would allow hospitals to minimize resource costs and maximize benefits. At the same time, patient hospitalization costs and the accompanying time burden for family members would be reduced, effectively reducing patient disease burden. The hospitalization cost for rural patients was lower than that for other patients, which may be related to the higher overall economic level of urban patients; rural patients tend to save more in the treatment process than urban patients. Moreover, the reimbursement rate for urban patients is mostly higher than that for rural patients. Additionally, unnecessary examinations or expensive drugs used in the treatment process could also result in higher hospitalization costs. However, owing to different medical insurance policies, the reimbursement rate of rural patients is low. In general, rural patients have a heavier economic burden. The total hospitalization cost for ethnic Zhuang patients was significantly lower than that for patients of other ethnicities. The reason for this trend is not completely understood but may be similar to that associated with the trend observed in rural patients; further study is needed in this area. Among China's ethnic minorities, the largest number is the Zhuang, with 65.63 percent of the rural population and 34.37 percent of the urban population [19]. But the per capita disposable income of urban residents is higher than that of rural residents (2.56 : 1) [20]. In addition, differences in economic development level and medical treatment level between urban and rural areas, as well as differences in living habits, eating habits, and disease spectrum [8], jointly lead to higher incidence and disease burden of nasopharyngeal cancer in rural patients than urban. So hospital management should be strengthened to ensure both treatment effect and the shortening of the average length of hospital stay. The economic burden of patients with nasopharyngeal carcinoma is particularly high for rural and ethnic Zhuang patients. It is recommended that the hospital management should adjust the hospitalization cost structure, control drug use proportions, reduce average hospitalization duration, and avoid excessive medical treatment to reduce the burden on patients [21].

The article "Demographics and Economic Burden of Nasopharyngeal Carcinoma Inpatients" was retracted in 2023. Reasons: signs of a paper mill; compromised peer review; unreliable results or conclusions.

This study was limited to the analysis of direct costs in the economic burden of patients; indirect and intangible costs were not quantified owing to the inability to obtain relevant data.

In conclusion, early diagnosis and treatment should be actively carried out to reduce the incidence of nasopharyngeal carcinoma, such as strengthening the science popularization education of nasopharyngeal carcinoma, popularizing EB virus antibody test [22, 23], conducting clinical trials of nasopharyngeal carcinoma vaccine, and improving the living habits and the quality of the ecological environment [3, 24], especially for rural, ethnic Zhuang, and males in the 40–49-year age group patients. The future research on nasopharyngeal carcinoma will focus on exploring the pathogenesis of nasopharyngeal carcinoma, improving the screening system [25], reducing the burden on patients, and formulating individualized treatment strategies, in order to further improve the survival rate and quality of life of patients with nasopharyngeal carcinoma.

## Figures and Tables

**Figure 1:** CONSORT diagram of the patient selection process.

**Figure 2:** Ethnic distribution of patients.

**Figure 3:** Scatter plot of the relationship between total hospitalization cost and age (a) and hospitalization days (b). *P* values were calculated with the Spearman rank correlation calculation.

**Table 1:** Gender comparison of nasopharyngeal carcinoma patients in different years.

Year	Male		Female		Total		Men-women ratio
	Cases	Constituent ratio (%)	Cases	Constituent ratio (%)	Cases	Constituent ratio (%)	
2012	146	72.64	55	27.36	201	5.39	2.65
2013	181	72.98	67	27.02	248	6.65	2.70
2014	357	75.64	115	24.36	472	12.67	3.10
2015	358	77.32	105	22.68	463	12.42	3.41
2016	356	75.91	113	24.09	469	12.58	3.15
2017	366	72.62	138	27.38	504	13.52	2.65
2018	314	72.85	117	27.15	431	11.57	2..68
2019	351	73.43	127	26.57	478	12.83	2.76
2020	336	72.89	125	27.11	461	12.37	2.69
Total	2765	74.03	962	25.97	3727	100	2.87

**Table 2:** Age distribution of patients.

Age group (years)	Male	Female	Total	Men-women ratio	Constituent ratio (%)
<20	24	12	36	2	0.97
20~	148	57	205	2.60	5.50
30~	526	217	743	2.42	19.93
40~	970	304	1274	3.19	34.18
50~	731	251	982	2.91	26.35
60~	309	108	417	2.86	11.19
70~	55	12	67	4.58	1.80
80~	2	1	3	2	0.08
Total	2765	962	3727	2.87	100

**Table 3:** Variation trend of average length of stay.

Year	Average length of stay (days)	Annual increment (days)	Link relative ratio (%)
2012	46.32 ± 20.55	—	—
2013	43.84 ± 20.11	-2.48	-5.35
2014	39.23 ± 23.76	-4.61	-10.52
2015	37.17 ± 24.86	-2.06	-5.25
2016	37.75 ± 23.25	0.58	1.56
2017	32.67 ± 22.97	-5.08	-13.46
2018	31.47 ± 24.63	-1.2	-3.67
2019	40.99 ± 15.34	9.52	30.25
2020	35.42 ± 16.75	-5.57	-13.59
Average value	38.32 ± 4.61	−1.36	-2.50

**Table 4:** Variation trend of hospitalization expenses.

Year	Hospitalization cost per case (yuan)	Annual increment (yuan)	Link relative ratio (%)
2012	54312.95	—	—
2013	63901.44	9588.49	17.65
2014	56635.44	-7266	-11.37
2015	55187.16	-1448.28	-2.55
2016	59009.9	3822.74	6.92
2017	59600.7	590.8	1.00
2018	57750.38	-1850.32	-3.10
2019	90443.44	32693.06	56.61
2020	85988.87	-4454.57	-4.93
Average value	64758.92	3959.49	7.53

**Table 5:** Analysis of partial factors influencing total hospitalization costs.

Factors	*N*	Hospitalization cost (yuan)	*P* value
Gender			
Female	962	76470.07 ± 42281.67	0.807
Male	2765	77305.90 ± 42954.43	
Ethnicity			
Han	2153	68800.63 ± 43354.23	≤0.001
Zhuang	1460	60624.60 ± 41663.67	
Others	114	68787.48 ± 40027.48	
Rural/urban			
Rural	2223	61454.37 ± 41559.61	≤0.001
Urban	1504	71720.99 ± 43815.87	

The article "Demographics and Economic Burden of Nasopharyngeal Carcinoma Inpatients" was retracted in 2023. Reasons: signs of a paper mill; compromised peer review; unreliable results or conclusions.

**Table 6:** Multiple linear regression analysis of hospitalization expenses.

Variable	*b*	SE	*b*′	*t*	*P*
Constant	3.992	0.011		373.311	≤0.001
Ethnic group	-0.019	0.008	-0.022	-2.204	0.028
Rural/urban	0.027	0.010	0.027	2.780	0.005
Length of stay	0.017	0.000	0.800	81.675	≤0.001

**Table 7:** Impact of comparison between rural and urban patients on total hospitalization costs.

Variable	*b*	SE	*b*′	*t*	*P*
Constant	4.698	0.012		381.648	≤0.001
Rural	-0.093	0.016	-0.095	-5.825	≤0.001
Urban	0				

## Data Availability

These data used to support the findings of this study are available from the corresponding author upon request.
